The article "An Exploratory Study on the Effects of Invisible Violence on Students' Mental Health in Physical Education" was published in 2022. Journal: J Environ Public Health.

# An Exploratory Study on the Effects of Invisible Violence on Students' Mental Health in Physical Education

**DOI:** 10.1155/2022/8349916

**Published:** 2022-09-12

**Authors:** Duan Liang, Ren Xiangjing

**Affiliations:** ^1^School of Physical Education, Shandong Sport University, Rizhao 276800, China; ^2^Physical Education Institute of Jimei University, Jimei University, Amoy 361021, China

## Abstract

Invisible violence in school physical education can negatively affect students' body and mind and is detrimental to students' sports cognition, sports participation, and sound personality cultivation and shaping. We analyze the manifestation and causes of invisible violence in physical education and propose a path to eliminate it, so as to improve the quality of school physical education and promote students' physical and mental health. In this study, 30 students were interviewed, relevant research data were collected, and coding and clustering were conducted using the rooting theory research method. The results of the study are as follows: Invisible violence in physical education is characterized by concealment, unconsciousness, and indirect harm. According to the 11 characteristics of invisible violence in physical education, invisible violence in physical education is classified as invisible behavioral violence, invisible verbal violence, and invisible discrimination violence. The root causes of invisible violence in physical education are physical education teachers' lack of understanding of the value of physical education, misplaced transfer of bad emotions and teaching. The root causes of invisible violence in physical education are teachers' lack of understanding of the value of physical education, misplaced emotions, and the wrong expression of teaching language. The three countermeasures to eliminate invisible violence in physical education are: reshaping physical education teachers' professional beliefs, improving physical education teachers' emotional self-management ability, and strengthening physical education teachers' oral expression ability.

## 1. Introduction

With the gradual improvement of laws, the change of educational philosophy, the soundness of school regulations, and the improvement of physical education teachers' comprehensive quality, explicit violence such as corporal punishment, beating, verbal abuse, and sexual assault committed by physical education teachers against students has been effectively managed, and the status of physical education discipline and the social image of physical education teachers have been enhanced [1]. Construction to the national level, reflecting the importance the state attaches to education and at the same time putting forward higher requirements for the professional conduct of teachers in the new era. Before that, the Ministry of Education issued the Code of Ethics for Teachers in Primary and Secondary Schools and the Code of Ethics for Teachers in Higher Education, which regulate the professional ethics of teachers in schools and colleges, providing a policy guarantee to better promote respect for teachers and create a good environment for educating people. Physical education is an important part of school education, and the purpose of school physical education is to improve the physical quality of students and promote their healthy physical and mental development. The period of school physical education is large; from preschool education to university sequence involves physical education [2]. The teaching of physical education in schools involves both the teaching of sports knowledge and the development of sports skills, which play an important role in the development of healthy exercise habits, the mastery of physical exercise knowledge and skills, and the enhancement of the physical fitness and health of students. Physical education teachers have a special way of teaching, which includes verbal explanation, physical demonstration, and correction of students' movements, along with verbal communication and physical guidance. It is found that due to the differences in students' individuality, which lead to the uneven mastery of students' physique, body type, and motor skills, it is difficult for physical education teachers to teach in a way or means that satisfies every student in the face of different situations, which will make some students with poor physique or fat body type struggle to practice and fail to complete the classroom teaching tasks, and teachers face students with a poor physical condition or poor motor foundation The teachers' intentional or unintentional discrimination and indifference in the face of students with poor physical condition or poor athletic foundation can easily cause students' frustration and make students' self-esteem hurt, which is not conducive to their learning of physical education knowledge and skills. It was found that although the phenomenon of explicit violence in school physical education is gradually decreasing, invisible violence such as indifference, discrimination, and neglect in verbal and behavioral violence exhibited by physical education teachers in physical education still exists to some extent [3]. If this undesirable phenomenon is not effectively curbed in school physical education, it will have a negative impact on students' body and mind, which is not conducive to students' sports cognition, sports participation, and sound personality development and shaping. This study used in-depth interviews to collect relevant research data, analyze the manifestation and causes of invisible violence in physical education, and propose a path to eliminate it, so as to achieve the purpose of improving the quality of physical education in schools and promoting students' physical and mental health.

The article "An Exploratory Study on the Effects of Invisible Violence on Students' Mental Health in Physical Education" was published in 2022. Journal: J Environ Public Health.

## 2. Literature Review

The teacher-led and student-led forms of teaching interaction in physical education areconducive to the dissemination of physical health knowledge and the learning of physical skills. Physical education is different from simple theoretical teaching in that, firstly, the teaching field is different; both the teaching environment is different; and the theoretical teaching environment is mostly classroom and the physical education environment is mostly outdoors. Secondly, the content of teaching is different. Theoretical teaching is mostly about the transmission of knowledge, while physical education includes both the transmission of physical exercise knowledge and the cultivation of sports skills. Finally, the learning mode is different. Theoretical learning is to memorize as the main body and mastery as the purpose, and physical education learning is to have direct physical participation experience as the main body and mastery of skills acts as the purpose [4].

In outdoor physical education, teachers organize appropriate formation through language to motivate students to participate in the learning of physical skills, and language exchange and communication become the prerequisite for physical education between teachers and students. Teachers prompt students on the main points of actions and problems through language, ask students about their practice experience, and students give feedback on their learning experience, which becomes an important part of physical education. But since students come from different places of origin, different learning and growing environments, and therefore different dialects and accents in different places, the accent or dialect of students in physical education can easily cause teachers to be geographically discriminatory [5]. Intentional or unconscious criticism of error correction by teachers in physical education can cause psychological frustration in some students with high self-esteem, resulting in low mood and a reduced interest in participating in sports [6]. Work and family are the places where teachers spend most of their time and energy, and family relationships affect teachers' emotional expression; teachers' emotions that are not well controlled in physical education will be poorly expressed in physical education, such as chaotic teaching organization, rough teaching actions, and unreasonable exercise, which will have a negative impact on students' physical and mental health and interest in learning sports [7]. Most physical education teachers are athletes with good physical quality and high motor skills, and they have high requirements for movement learning and physical quality, and when students fail to meet the required standards, teachers show dissatisfaction with their attitudes and body language, which can easily make students lose their emotions, lower their self-identity, and negatively affect their interest in physical exercise [8]. In physical education, due to the variability of the student population, there are obese students who move more slowly in running and jumping and cannot complete their movements flexibly; short students, who cannot complete their tasks in strength exercises; and timid female students, who are afraid to engage in strenuous exercises, all of which are easily treated with indifference and neglected by physical education teachers and affect the learning of physical skills and the development of physical and mental health of students [9]. Existing studies in the literature dealing with the adverse factors that exist in school physical education that affect the development of physical education and the subjective factors that physical education teachers tend to ignore provide a theoretical basis for the study of implicit violence in school physical education. However, the existing literature is inconclusive as to what forms of hidden violence exist in physical education and what characteristics and behavioral manifestations affect the healthy development of physical education, so it is of great theoretical and practical significance to extract the manifestations of hidden violence to analyze its causal characteristics and propose a path to solve it through a research method rooted in theory.

The article "An Exploratory Study on the Effects of Invisible Violence on Students' Mental Health in Physical Education" was published in 2022. Journal: J Environ Public Health.

## 3. Research Methods

### 3.1. In-Depth Interview Method

The in-depth interview method is an unstructured qualitative research method [10] in which trained facilitators talk to recruited students in an unstructured, naturalistic format, and 30 interview volunteers were recruited from June to August 2021 in a stance sampling of university, secondary, and elementary school students, sorted using the sequential method, and each interviewer was snowballed on the invisible influences of violence in school physical education Factors were deeply explored and collected. Before conducting the interviews, the interviewees were first informed of the purpose of the interview, without the appearance of names or schools, and they signed a privacy agreement with the consent of the interviewees. The moderator controlled the rhythm and orientation of the interview, focusing on the typical incidents encountered during physical education classes and physical education teaching to provide a specific description of the words or behaviors of physical education teachers who implemented words or behaviors that did not gain the psychological approval of the students and had an excessive impact on their emotional and psychological tolerance and thus produced harm during the teaching of art and theory classes, based on the interviewees' perceptions and evaluations. In the case of unclear expressions or ambiguous concepts, the moderator communicated with the interviewees and accurately recorded the accuracy of the information expressed by the interviewees, and the length of the interview was 45–60 minutes per person, totaling 23 hours.

### 3.2. Rooted Theory Research Method

The rooted theory research method follows practice and is not based on existing theories. The researcher generally has no theoretical assumptions before the study begins, starts directly from actual observations, summarizes empirical generalizations from primary sources, and then rises to a systematic theory, which is a bottom-up approach to theory construction [11]. The audio recordings of 30 interviewees were first organized, and the 23 hours of interview recordings were converted into text documents, extracting a total of 37596 words of interview text and 8643 words of this memo. Then open coding was performed word-by-word, sentence-by-sentence, and paragraph-by-paragraph so that the concepts were naturally presented and the categories and concepts were extracted. In the coding process, sensitivity to theory was maintained, the connotation and extension of the concepts were repeatedly compared and deliberated, and the subordination was determined. Based on the open coding, the extracted concepts and categories were clustered and coded to establish connections between concepts and categories and to cluster concepts and categories to make the categories and dimensions specific. Finally, from the perspectives of physical education, education, psychology, and management, we use analogies, deductions, inductions, analyses, and other logical methods to summarize and conclude the manifestations, causes, and countermeasures to eliminate invisible violence in school physical education.

## 4. Research Results and Analysis

### 4.1. Definition of the Concept of Invisible Violence in Physical Education

Violence refers to rape against the person and property of others and can be divided into verbal violence and behavioral violence. Verbal violence is mainly carried out by “insults” and “aggressive language” with the nature of “prejudicial language” [12]; behavioral violence is mainly manifested by physical conflict, corporal punishment, and disguised corporal punishment [13]. Behavioral violence is mainly manifested by physical conflict, corporal punishment, disguised corporal punishment, etc. [13]. The concept of “invisible violence” proposed in this study is closer to the expressions of “cold violence,” “soft violence,” “mental violence,” and “psychological violence,” “Psychological violence,” and so on. Combining the previous research results and the special nature of physical education activities, this study defines “invisible violence in physical education” as the words or behaviors of physical education teachers that do not gain students' psychological recognition and have an excessive impact on their emotional and psychological capacity, thus producing harm. The French sociologist Pierre Bourdieu proposed the concept of “field”, which defines a field as a network or a configuration of objective relations between positions, which are objectively limited [14]. In this study, the field of physical education is limited to the locations or spaces directly related to the implementation of physical education, such as physical education technology courses, physical education theory courses, and physical education tests.

The article "An Exploratory Study on the Effects of Invisible Violence on Students' Mental Health in Physical Education" was published in 2022. Journal: J Environ Public Health.

### 4.2. Content Extraction and Coding of Invisible Violence in Physical Education

Firstly, the statements were stripped, and the statements related to the main idea of this paper were selected for word-by-word text transcription; secondly, the obtained text was coded line by line, and the coding rule was “interview time + scene + interviewer code + number of lines.” For example, finally, in the process of data analysis, we used the thematic analysis method, repeatedly reading the statements, extracting them according to the contextual meaning and the theme of expression, and gradually focusing the open coding of the statements to obtain the symbolic codes (see Table 1), merging the symbolic codes according to the attributes to form The keywords such as “indifference” were formed. The interview text was coded word-by-word and sentence-by-sentence, and when it was carried out to the 22nd person, no new categories were generated, and when the coding of 8 more people was carried out, no new categories were generated, so it was judged as theoretical saturation.

### 4.3. Performance of Invisible Violence in Physical Education

According to the key event interviews of the interviewees of invisible violence in physical education, the content of the event was analyzed for its semantic and connotation of invisible violence for open coding, 46 categories were extracted, and the connotation and extension of the 46 categories were clustered to refine 11 terms with the characteristics of invisible violence. Accordingly, the 11 relevant invisible violence features of invisible violence were categorized into three areas: invisible behavioral violence, invisible verbal violence, and invisible discrimination violence (see Table 2).

The article "An Exploratory Study on the Effects of Invisible Violence on Students' Mental Health in Physical Education" was published in 2022. Journal: J Environ Public Health.

Invisible behavioral violence is manifested by the physical education teacher's intentional or unintentional indifference, neglect, and unfair treatment of students, and this indifference or neglect is directed to the psychological level; this “no one in sight” situation or bland response or no response to students affects the public image of physical education teachers and students' perceptions of physical education, making students feel subjected to. This “no one” situation or a bland or no response to students affects the public image of physical education teachers and students' perceptions of physical education, making students feel coldly treated, generating interpersonal frustration, leading to lower self-evaluation, and causing bias in students' perceptions of teacher-student relationships in physical education and causing hidden psychological harm to students [15]. At the same time, if physical education teachers lack respect for teaching and students and fail to reflect the educational concept of “teaching at random” in physical education, it will make individual students have negative psychological experiences in the process of participating in sports, which is not conducive to the construction of motor habits and motor abilities.

Invisible verbal violence is manifested as negative language and verbal coercion in physical education, mainly from emotion, power, or traditional teacher-student moral pressure, so that students will have pressure transmission, resulting in increased psychological pressure, negative emotions, and a sense of damage to the personality and dignity of students. Physical education teachers who use excessive negative language and verbal coercion are also responded to by students. Response strategies are retaliatory in nature. For example, the teacher is given a lower grade during the evaluation of their teaching. In physical education, physical education teachers also have emotional changes and use certain channels to vent their emotions, i.e., when they communicate with students or talk about them after class, they use and understand individual words differently and give derogatory comments, some of which do not reach a significant magnitude to determine whether there is a certain amount of verbal harassment or aggression, which can also cause students to be “colored” in physical education. Some of these comments, although not of a significant magnitude, do not determine whether there is a certain amount of verbal harassment or aggression, but can also cause students to be viewed through “colored glasses” in physical education, resulting in a misunderstanding in communication [15].

The article "An Exploratory Study on the Effects of Invisible Violence on Students' Mental Health in Physical Education" was published in 2022. Journal: J Environ Public Health.

Invisible discrimination violence manifests itself as a degree of “differentiation” and “labeling” in the field of physical education, but mostly as potential mental discrimination. Cultural differences, especially significant linguistic differences, are important factors in the formation of geographical discrimination chains. Because women are disadvantaged in terms of physiological functions and athletic qualities, school sports facilities are designed for male-dominated programs, and the settings and specifications of venues and equipment are largely based on male needs [15]. As a result, “gender stereotyping and gender bias in extracurricular sports participation” often occur in physical education [16]. The body is not only a physical body in a physiological sense but also a body in a culturally competent symbolic sense, so discrimination against the body actually devalues the whole of life at a practical level [17]. Physical education teachers have different degrees of invisible body discrimination due to the existence of internal misjudgments due to differences in external characteristics of students such as height, physical ability, size, and appearance.

### 4.4. Characteristics of Invisible Violence in Physical Education

First is invisibility. Institutional constraints are an important reason for the generation of invisible violence in physical education, which lies in the fact that physical education also involves the operation of power [18], due to the institutional cultural constraints, and thus there are some irrational behaviors that are more hidden and not directly or explicitly mentioned by the relevant laws and regulations as well as the teaching system during the implementation of physical education activities.

Second is unconsciousness. Influenced by the traditional Chinese Confucian culture of “dignity of the teacher” and “respect for the teacher” and other ethics, the power of teachers and students in the process of physical education is still not equal. Physical education, which is the carrier of the power system, has become a place where physical education teachers are prone to violence or invisible violence, and the unconscious words and actions of physical education teachers in physical education activities have caused psychological conflicts and discomfort between teachers and students.

The article "An Exploratory Study on the Effects of Invisible Violence on Students' Mental Health in Physical Education" was published in 2022. Journal: J Environ Public Health.

Third is indirect injuriousness. The negative experiences of adolescents in the process of physical activity directly lead to a lack of motivation or interruption of their sports participation [19], and although invisible violence in physical education does not cause direct physical harm to students, these behaviors can cause adverse psychological experiences for students, affecting teacher-student relationships, teaching effectiveness, and damaging teachers' images.

### 4.5. Effects of Invisible Violence in Physical Education on Students' Psychological Health

The purpose of school physical education is to improve students' physical and mental health, and the learning of physical education knowledge and skills is explicit and can be objectively evaluated through external performance. For example, the completion degree and number of pull-ups can be reliably counted and measured, and the mastery of physical education knowledge can be evaluated through tests. However, the behavior, language, and discrimination that teachers intentionally or unintentionally perform on students in physical education implicit violence injuries are persistent and insidious. Implicit verbal violence hurts students' self-esteem, affects their self-perception and self-evaluation, makes them think that they are not suitable for sports, and is detrimental to their learning of physical education knowledge and skills; implicit discriminatory violence makes students suffer from discrimination and indifference, which can make them afraid to cooperate with other students in learning, for fear of affecting the performance of other students or groups, thus making them autistic or depressed. Implicit behavioral violence causes students to receive physical and psychological harm, generating psychological shadows and fears, fearing, and rejecting participation in sports.

## 5. Discussion

### 5.1. Physical Education Teachers' Lack of Understanding of the Value of Physical Education Induces Invisible Violence

“Physical literacy” comprehensive education is the mainstream of current physical education, and in 2016, the General Office of the State Council issued the Opinions on Strengthening School Sports for the Comprehensive Development of Students' Physical and Mental Health (i.e., “Document 27”), which for the first time from the national level once again In 2016, the General Office of the State Council issued the Opinions on Strengthening School Physical Education for the Overall Development of Students' Physical and Mental Health (“Document 27”), which was the first time that the overall improvement of students' physical education was explicitly proposed as one of the basic principles of future school physical education in China [20]. However, due to the influence of traditional physical education ideology and a lack of in-depth understanding of the value of physical education, physical education teachers still adhere to a single physical education to a large extent, which inevitably produces two opposing phenomena in physical education: first, physical education is only focused on the body, failing to pay attention to the role of physical education on students' comprehensive literacy; and second, long-term physical education is the main line, obscuring the educational value of physical education. First, physical education is only for the body and fails to pay attention to the role of physical education in students' comprehensive literacy, which has long been the main line of physical education, obscuring the educational value of physical education. Second, “disciplining” students' bodies is very likely to trigger students' rebellious mentality. Both of these phenomena are likely to lead to teachers' wrong words or behaviors and produce a certain degree of invisible harm.

The article "An Exploratory Study on the Effects of Invisible Violence on Students' Mental Health in Physical Education" was published in 2022. Journal: J Environ Public Health.

### 5.2. Invisible Violence Is Induced by the Misplaced Transfer of Bad Emotions of Physical Education Teachers

Hargreaves identified teacher emotions as one of the most neglected dimensions of educational change [21]. In exploring the causes of the phenomenon of invisible violence in physical education, it is also important to note the behavioral logic behind teachers' perpetration of invisible violence. The numerous elements, links, and frequent interactions in physical education directly affect teachers' emotional stability, generating adverse emotions resulting in a loss of confidence, a sense of control, and a reduced sense of motivation to achieve, triggering teachers' emotional catharsis. In addition, physical education teachers are prone to burnout in a state of physical and psychological exhaustion, which affects their emotional commitment to teaching and invisible violence such as indifference, neglect, and discrimination. The misplaced transfer of undesirable emotions is an important logical starting point for analyzing invisible violence in physical education, which largely guides physical education teachers' thinking, judgment, decision-making, and actions. The issue of physical education teachers' emotions and the physical education behaviors they spawn is often overlooked by the teachers themselves. It can be seen that the invisible violence in physical education is due to the misdirected cathartic process of physical education teachers' placing their bad emotions in physical education, which leads to misplaced words and actions in the process of physical education.

The article "An Exploratory Study on the Effects of Invisible Violence on Students' Mental Health in Physical Education" was published in 2022. Journal: J Environ Public Health.

### 5.3. Invisible Violence Is Induced by the Wrong Language Expressions of Physical Education Teachers

Physical education is not only about teaching by example but also about teaching by word, so the ability of physical education teachers to use language is an important guarantee for the implementation of physical education. Physical education teachers have a certain amount of dominant discursive power as a result of the power given to them by the educational system and cultural traditions. The use of discursive power by physical education teachers includes the professionalization of physical education teachers to explain, instruct, demand, and discuss, as well as to criticize within the prescriptive scope of education. If teachers misunderstand and use this power to assert their authority and criticize or evaluate students beyond educational prescriptiveness, they are more likely to misuse discourse and engage in invisible verbal violence. The damage to students' minds from invisible verbal violence is often not something that can be quickly bridged over time and is long-lasting [22].

### 5.4. Remodeling Physical Education Teachers' Professional Beliefs Can Avoid Hidden Violence

Since the current important guiding idea of physical literacy has introduced physical education as a “psychomotor learning goal in the affective and cognitive domains” [23], the value of physical education should not only be satisfied with the basic functions of developing physical fitness and motor skills of students but should also include the cultivation and enhancement of students' physical literacy in the scope of physical education. In other words, the relationship between teachers and students in physical education is not the oppressive relationship of training in physical fitness improvement but the cooperative relationship of improving physical literacy. Physical education teachers should change the traditional physical education concept that physical education is only located in human “body” education and cooperate with students to complete diversified physical education tasks so as to avoid the emergence of invisible violence in physical education.

### 5.5. Improving Physical Education Teachers' Emotion Management Ability Can Avoid Hidden Violence

Emotion management ability is a skill that involves awareness of one's own emotions and the emotions of others, as well as developing the ability to manage emotions. The process of physical education involves a lot of emotional work, and physical education teachers are the leaders and implementers of physical education work, so they need to treat, understand and recognize their own emotions correctly; have the ability to control their own emotions;adopt appropriate ways to express their emotions; and carry out rational control, cognitive adjustment, and reasonable catharsis. Therefore, physical education teachers should have good emotional self-management ability when instructing or criticizing students in physical education and avoid using stressful words and actions.

The article "An Exploratory Study on the Effects of Invisible Violence on Students' Mental Health in Physical Education" was published in 2022. Journal: J Environ Public Health.

### 5.6. Strengthening Physical Education Teachers' Oral Expression Ability Can Avoid Hidden Violence

Physical education teachers need to use instructive and evaluative language in the process of physical education to speak about students' mastery of physical skills. If excessive blaming, complaining, and criticism occur when instructing and evaluating students' shortcomings or mistakes in the process of mastering physical skills, it can cause verbal misuse caused by emotional expression. Some of the language misuses that occur in physical education teachers can be classified as inadvertent. The probability of such language misuse can be reduced by improving physical education teachers' language literacy, avoiding unconscious and invisible verbal violence as much as possible, and minimizing invisible verbal harm to students. Therefore, physical education teachers should strengthen their oral expression training and improve their ability to use oral expression and use it.

## 6. Conclusion

Invisible violence in physical education is prevalent in physical education activities, and it has the characteristics of concealment, unconsciousness, and indirect harm. According to the 11 characteristics of invisible violence in physical education, invisible violence in physical education is divided into invisible behavioral violence, invisible verbal violence, and invisible discrimination violence. Invisible behavioral violence makes students suffer from cold treatment, frustration, and lower self-evaluation; invisible verbal violence increases students' psychological pressure and damages their self-perception of personality and dignity; invisible discrimination violence belongs to potential mental discrimination, and physical, gender, and geographical discrimination are important triggers for the formation of an invisible discrimination chain.

The root causes of invisible violence in physical education are physical education teachers' lack of understanding of the value of physical education, misplaced transfer of bad emotions, and wrong expression of teaching language; the countermeasures to eliminate invisible violence in physical education are: reshaping physical education teachers' professional beliefs; improving physical education teachers' emotional self-management ability; and strengthening physical education teachers' oral expression ability.

The article "An Exploratory Study on the Effects of Invisible Violence on Students' Mental Health in Physical Education" was published in 2022. Journal: J Environ Public Health.

## Figures and Tables

**Table 1:** Example of analysis of the set of invisible violent symbols in physical education.

Original Recording	Symbol	Property	Number
I did not want to take a soccer class, but I could not take the class I liked, so I had to take soccer, and I had never played soccer before, so I did not have much foundation. But the teacher did not care about our situation in class, just taught according to his method, and did not care much about the poor foundation, so he went to play a game with those who had a good foundation	Forced to	Indifferent treatment	20210609A01L01
	Disliked		20210609A01L02
	No exposure		20210609A01L03
	No foundation		20210609A01L04
	No matter	Neglect	20210609A01L05
	Method		20210609A01L06
	No matter		20210609A01L07
	Good foundation		20210609A01L08

**Table 2:** Composition of invisible violence in physical education.

Dimensionality	Behavioral properties			
Invisible behavioral violence	Indifferent treatment	Intentional or unintentional neglect		Unfair pinging

Invisible verbal violence	Negative language	Verbal coercion		Language ambiguity
	Verbal harassment		Backbiting	

Invisible discrimination violence	Sexism	Geographical discrimination		Physical discrimination

## Data Availability

All the data included in this study are available upon reasonable request to the corresponding author.
